# Radiation Dose Exposure to Patients During Transcatheter Patent Ductus Arteriosus Closure via the Arterial Route

**DOI:** 10.7759/cureus.30685

**Published:** 2022-10-25

**Authors:** Abdulkader M Alsharif, Yasser A Bhat, Abdulrahman Al Mesned, Abdullah Al Qwaee, Ali Al Akhfash

**Affiliations:** 1 Pediatric Cardiology, Prince Sultan Cardiac Center - Qassim, Buraydah, SAU; 2 Cardiovascular Sciences, Sapienza Università di Roma, Rome, ITA

**Keywords:** patent ductus arteriosus closure, radiation dose, intervention pediatric cardiology, cath lab, radiation dose reduction

## Abstract

Objective

This study aims to evaluate the radiation dose for transcatheter patent ductus arteriosus (PDA) via the arterial route and compare it with previously published benchmarks.

Background

Exposure to radiation in the catheterization lab can cause skin injury and cancer in the long run, especially in pediatric patients with complex heart conditions, which necessitate serial catheterizations. Therefore, measuring the patient radiation dose and establishing a benchmark for each cardiac interventional procedure is essential.

Material and methods

In this prospective study, 34 patients with transcatheter patent ductus arteriosus closure via an arterial route were included. Patients who had silent PDAs, no left heart dilatation and PDA size of less than 2mm had PDA closed via an arterial route. All the study group patients received an Amplatzer duct occluder II-additional size device (St. Jude Medical Corp, St. Paul, MN) using biplane flat-panel fluoroscopy equipment adjusted in accordance with the pediatric parameters. Patients' dose area product, air kerma and fluoroscopy time were recorded in the catheterization lab and finally compared with internationally published reference data.

Results

Of 73 patients who had transcatheter patent ductus arteriosus closure between April 2021 to December 2021, 34 patients who had a PDA closure via an arterial route were enrolled. The median age and weight were 11.5 (4-168) months and 10.5 (6-31) kg. Twenty-one (61.8%) were males, and 13 (38.2%) were males. The median radiation dose parameters were as follows: air kerma 11 (3-42) milliGray, dose area product 131 (33-443) microGray per m^2^, median dose area product indexed to weight 12 (1-48) microGray m^2^ per kg, fluoroscopy time 2 (2-4) min and frame rate 15 (7.5-15) frames per second. Due to many factors, our radiation dose parameters were less than internationally published reference values for transcatheter PDA closure.

Conclusion

Patient selection, detailed pre-catheterization echocardiography and procedure planning are essential for accomplishing device closure of PDA with a significant reduction in radiation dose. Hemodynamic assessment in the catheterization lab is unnecessary for most PDA patients. Additionally, a next-generation imaging platform equipped with flat-panel detectors and adjusted for pediatric settings and a fluoro recording option can be used to reduce radiation exposure.

## Introduction

Diagnostic radiological examinations in infants and children present a higher risk of developing cancer per unit of radiation dose than in adults. The increased risk in children is due to their longer life expectancy, leaving more time for the harmful effects of radiation to manifest. Also, developing organs and tissues are more sensitive to the effects of radiation [1]. Moreover, children with complex congenital heart disease are often catheterized repeatedly, so the risk of radiation-induced cancer is higher in children than in adults [2]. Consequently, maintaining radiation doses to patients and staff as low as reasonably achievable (ALARA) is strongly supported by the Society for Pediatric Radiology, especially when using procedures and modalities involving higher radiation doses, such as pediatric CT and fluoroscopic exams [3]. Children are exposed to high radiation levels during cardiac procedures but with a considerable variation in radiation dose; therefore, particular attention should be given to radiation dosimetry during cardiac catheterization [4-5]. Reference data on radiation exposure for congenital cardiac catheterization is difficult to obtain due to the high complexity of procedures affected by the underlying pathology and the type and quality of prior imaging. Differences in age, size, equipment specifications and interventionists' skills add to this heterogeneity [6]. As a result, radiation dose measurements released for reference and comparison between pediatric cardiac catheterization procedures are rare [7]. The study aims to analyze the radiation dose, especially dose area product (DAP) and air kerma, for closing the patent ductus arteriosus by retrograde approach and compare it with the previously published benchmarks [6-9].

## Materials and methods

In a prospective study between April 2021 and December 2021, 34 patients with patent ductus arteriosus (PDA) catheter closure via an arterial route participated. The study was carried out in the Department of Pediatric Cardiology, Prince Sultan Cardiac Center, Qassim and approved by the institutional review board. Although the patients had PDA closed via antegrade and retrograde approaches, patients who had PDA device closure via retrograde approach were included. Patients were selected for transcatheter PDA closure based on clinical and echocardiographic evaluation at the outpatient clinic. Patients who had silent PDAs, no left heart dilatation and PDA size less than 2mm had PDA closed via an arterial route (femoral artery). None of the patients had a hemodynamic evaluation in the catheterization laboratory before device placement. All the study group patients received an Amplatzer duct occluder II-additional size device (St. Jude Medical Corp, St. Paul, MN) via a four French Amplatzer^TM^ TorqVue^TM ^Low Profile Delivery System (AGA Medical Corporation, North Plymouth, MN). (Table 1)

**Table 1:** Size of Amplatzer duct occluder II- additional size implanted among the patient population N, number of patients; %, percentage

Device size (mm)	N (%)
4mm x 4mm	16 (47.0)
4mm x 6mm	6 (17.6)
5mm x 6mm	5 (14.7)
5mm x 4mm	5 (14.7)
5mm x 2mm	1 (2.9)
4mm x 2mm	1 (2.9)

We operate Siemens Artis Zee (Siemens Shanghai Medical Equipment Ltd. 278 Zhou Zhu Road 201318 Shanghai China) biplane flat-panel fluoroscopy equipment in the catheterization laboratory. The machine has been adjusted in accordance with the pediatric parameters (Table 2).

**Table 2:** Imaging platform parameters for fluoro in our catheterization laboratory. Kg kilogram; cm centimetres; mA milliamperes; kV kilovolts; mm millimetre

System setting (for fluoro)	Weight < 6 Kg	Weight 6-20 Kg
Flat-panel detector	20 cm x 20 cm	20 cm x 20 cm
Current	100 mA	100 mA
Voltage	70 kV	70 kV
Pulses per second	10	15
Copper filtration	0.3 mm	0.3 mm
Magnification	10-25 cm	10-25 cm

Furthermore, the machine is used exclusively for pediatric cardiac patients. In addition, ALARA concepts have been applied to minimize radiation exposure. The control room computing system displays patients' radiation dose information, dose area product (DAP), air kerma, and fluoroscopy time. Patients' demographic characteristics and radiation dose information were recorded in the format created in Google Forms. A Google spreadsheet was generated, data analyzed, and median DAP, air kerma and fluoroscopy time were calculated. Finally, the radiation dose exposure for PDA catheter closure via retrograde approach was compared with previously published reference values.

Data management and analysis

The data was stored and compiled in Google forms and a Google spreadsheet. The analysis was conducted using statistical software embedded in a Google spreadsheet, and the median DAP, air kerma and fluoroscopy time were calculated.

## Results

A total of 73 patients had transcatheter closure of PDA at our centre during the study period. Only 34 patients with transcatheter PDA closure via an arterial route were enrolled. The rest of the 39 patients who had PDA closed by venous route were excluded. Twenty-one (61.8%) were males, and 13 (38.2%) were females. The demographic characteristics are shown in Table 3. 

**Table 3:** Demographic characteristics of the patients

Variable	Median	Range
Age (months)	11.5	4-168
Weight (Kilograms)	10.5	6-31
Height (centimeters)	71.5	60-160

Twelve patients (35.3%) were over one year of age, and the remainder, 22 (64.7%), were under one year of age. Most of our patients weighed less than 20 kg; only two had a weight greater than 20 kg. All had a successful PDA device closure using an Amplatzer duct occluder II - additional size via an arterial route without significant adverse events. The radiation dose for the patient population is shown in Table 4.

**Table 4:** Radiation exposure dose to the patient population mGy: milli Gray; DAP: dose area product; mcGy/m2: micro Gray per square metre; fpm: frame per minute

Parameter	Median	Range
Air kerma (mGy)	11	3-42
DAP (mcGy/m^2^)	131	33-443
DAP/weight (mcGy/m^2^/Kg)	12	1-48
Fluoro time (min)	2	2-4
Frame rate (fpm)	15	7.5-15

Air kerma, DAP, DAP/kg and fluoroscopy time were expressed as median and ranges. Median air kerma, DAP, DAP/kg and fluoroscopy time were calculated for ages under one year and over one year. The radiation dose was then estimated based on age (Table 5).

**Table 5:** Air kerma (mGy), DAP (mcGy/m2), DAP/Kg (mcGy/m2/Kg) and fluoro time (min) stratified according to age group DAP: dose area product; mcGy/m2: micro Gray per square metre

	Age	
	Equal and less than one year	> one year
N (%)	22 (64.7)	12 (35.3)
Median air kerma	8	20
Median DAP	146	116
Median DAP/Kg	11	13
Median fluoro time	2	4

Finally, air kerma, DAP and fluoroscopy time were compared to published international reference studies [6-9] (Table 6).

**Table 6:** Comparisons of radiation doses with internationally published benchmarks

	Air Kerma (mGy)		DAP (mGy M2)		Fluoro time (min)	
	Median	Range	Median	Range	Median	Range
This study <20 Kg	9.5	3-42	131	33-443	2	2-4
Lamers et al. [8] patients < 20 kg	28	24–62	199	104–402	8.5	6–12
Glatz et al. [9] 5–12.5 kg	62	40–86	263	178–353	10.5	8–13
Our patients < one year old	8	3-42	146	33-443	2	2-4
Ghelani et al. [6] < one year old	76	65–90	500	400–600	15	13-16
Cevallos et al. [7] < one year	59	53-67	323	268-370	16	15-18

## Discussion

We analyzed DAP, air kerma, and fluoroscopic time in 34 patients with PDA closed by retrograde catheterization. Our patients were significantly less exposed to radiation than previously published baseline data [6-9]. The lower radiation dose exposure in our patient group could have been because of many reasons: (1) our machine has a save fluoro option, and the interventionists did not use cine-angiography for PDA device closure, (2) the machine is adjusted for pediatric settings, (3) the machine is equipped with a flat-panel detector, (4) we do not do a hemodynamic study as almost all the patients who had PDA closed by arterial route have tiny or small PDAs. Lamers et al. [8] described the dose reduction capabilities of a next-generation imaging system and documented a 60-70% decrease in DAP and air kerma in patients with PDA closed by the transcatheter method using fluoroscopic equipment adjusted to pediatric settings. In addition, they used the air gap technique and removed the anti-scatter grid. Although we did not use the air-gap technique and retained the anti-scatter grid, the DAP, air kerma, and fluoro time in our patient group were less than those of Lamers et al. [8].

While most fluoroscopes can automatically provide good image quality to infants, toddlers and young children, excessive radiation dose levels can result from imaging device design deficiencies or improper configuration of equipment capabilities when imaging small body areas. Essential design features and configuration options during the installation and clinical use of the imaging device can enhance image quality and reduce radiation exposure levels in pediatric patients [10]. Lamers et al. [8] compared the radiation dose between two different imaging systems adjusted to adult and pediatric parameters for the same procedure (transcatheter PDA closure). The study found a significant reduction in radiation dosage for the imaging system dedicated to pediatric patients and adjusted for pediatric parameters. Our centre has a cardiac catheterization laboratory dedicated to pediatric cardiac patients. Due to limited resources, it is common to use the adult catheterization laboratory for pediatric cardiac procedures, especially in developing countries, exposing the patients to an increased radiation burden. Patients with small or tiny PDAs were selected for transcatheter closure via an arterial route after a detailed assessment at the outpatient clinic. The authors demonstrated in another study [11] that hemodynamic catheterization assessment might not be required in clinically silent PDAs. As a result, transcatheter closure of the small/tiny PDA without hemodynamic evaluation may significantly reduce the radiation dose. Next-generation fluoroscopic devices are equipped with flat-panel detectors.

Using a flat panel system could account for reducing radiation exposure in our patients. The new flat panel system offers performance at lower dose levels and enhanced image quality and therefore seems to be a more appropriate technique for pediatric fluoroscopy than image-intensifier systems [12]. The cine angiogram is an essential contributor to the radiation dose, and the number of cine angiograms must be limited in a pediatric catheterization laboratory [13]. Because our fluoro unit has a save fluoro option, we perform the aortogram and take measurements on the stored fluoro. We do not do cine angiograms for patients with transcatheter PDA closure via an arterial route. That is another way to reduce our patients' exposure to radiation. Next-generation machines have a store fluoro option that experienced interventionists can utilize to limit the number of cine angiograms in the pediatric cardiac catheterization laboratory. Finally, the ease of use and the author's experience with the Amplatzer duct occluder II-additional size device could reduce the radiation dose.

Limitations

While this is a single-establishment study with a small sample size, this article provides primary data for future research efforts. This information will help estimate radiation dosage in patients with transcatheter PDA closure via an arterial route. Due to the small sample size, we could not stratify patients beyond one year in different age groups compared to internationally published baseline studies.

## Conclusions

Transcatheter PDA closure via the arterial route can be achieved with a significant decrease in radiation dose. Patient selection, detailed pre-intervention echocardiography and procedure planning are essential for accomplishing device closure of PDA with a significant reduction in radiation dosage. Hemodynamic evaluation in a catheterization laboratory is not required for most patients with PDA. Moreover, a new generation imaging platform equipped with flat-panel detectors adjusted for pediatric parameters will substantially reduce radiation. Additionally, a fluoro recording option can be used depending on the interventionist's expertise to mitigate further radiation exposure.
